# Paediatric Dupuytren’s Disease in a Child of Indian Ethnicity: A Case Report and Literature Review

**DOI:** 10.7759/cureus.20434

**Published:** 2021-12-15

**Authors:** Suzanne M Beecher, Quentin Jeantet, Kevin J Cronin

**Affiliations:** 1 Department of Plastic and Reconstructive Surgery, Children's Health Ireland an Temple Street, Dublin, IRL; 2 Department of Plastic and Reconstructive Surgery, Mater Misericordiae Hospital, Dublin, IRL; 3 Department of Plastic and Reconstructive Surgery, Children’s Health Ireland at Temple Street, Dublin, IRL

**Keywords:** interphalangeal joint, dupuytren’s disease, paediatric, child, joint contracture

## Abstract

Paediatric Dupuytren’s disease is a very rare clinical entity. Dupuytren’s disease has preponderance to older males of Celtic heritage. We present a case of Dupuytren’s disease in an eight-year-old boy of Indian ethnicity who presented with a progressive flexion contracture of his right ring finger for a duration of six months. On examination, he had an isolated 60-degree flexion contracture of the proximal interphalangeal joint with thickening of the skin and subcutaneous tissues. This was consistent with Dupuytren’s cord and contracture. He proceeded to theatre for a dermofasciectomy, with subsequent histological confirmation of Dupuytren’s disease. We performed a review of the literature and identified 21 reported cases of Dupuytren’s disease affecting the hand in the paediatric population. This is a rare report of Dupuytren’s disease affecting a child of Indian ethnicity.

## Introduction

There are multiple causes of flexion contracture of a digit in the paediatric population. Common presentations include a post-traumatic flexion contracture, with soft tissue or bony injury, or congenital causes such as camptodactyly or trigger finger. In this study, we present an unusual case of Dupuytren’s disease affecting an eight-year-old boy. Dupuytren’s disease is a fibroproliferative disorder that affects the palmar fascia. It is an autosomal dominant condition with variable penetrance. It has a preponderance for older men of Celtic heritage [1]. Whilst rare, Dupuytren’s disease can occur in adults of Indian ethnicity. It has a similar presentation and clinical course to Caucasian patients [2].

This is a report of a case of paediatric Dupuytren’s disease in a child of Indian ethnicity. In this study, we discuss the clinical presentation and management and highlight it as a rare but potential cause of flexion contracture in the paediatric population. We also aimed to perform a review of the literature to ascertain if similar cases have been encountered elsewhere.

## Case presentation

An eight-year-old boy of Indian ethnicity was referred to our plastic surgery service with a swelling over the volar aspect of his right ring finger. It was present for approximately six months. Over the previous two months, he became unable to fully extend the proximal interphalangeal joint. There was no associated pain or other symptoms. There was no history of trauma to the area. There was no family history of Dupuytren’s disease.

On examination, there was a palpable firm swelling superficial to the tendons with an associated skin pit. He had a flexion deformity of 60 degrees at the proximal interphalangeal joint that was not correctable with passive extension (Figure 1).

**Figure 1:** Flexion contracture right ring finger.

Ultrasound revealed soft tissue fibrosis superficial to the flexor sheath.

Dermofasciectomy was performed under general anaesthetic and tourniquet control. The disease was excised, including the overlying skin, with preservation of the neurovascular bundles (Figure 2).

**Figure 2:** Intra-operative image of excision of skin and underlying fibrous tissue.

Full passive extension of the digit was achieved. The defect was reconstructed with a full-thickness graft. The hand was placed in a volar resting, forearm-based back slab, with the metacarpo-phalangeal joint (MCPJ) at 15 degrees of flexion and the proximal interphalangeal joint (PIPJ) and distal interphalangeal joint (DIPJ) in extension. He was discharged home that day.

The patient was reviewed one week post-operatively. There was a full graft take. Gentle physiotherapy was commenced and a custom-made thermoplastic splint was made to keep the digit in extension when not exercising. Histopathological examination of the resected tissue confirmed the diagnosis of Dupuytren’s disease.

## Discussion

In this case, we report a very rare cause of digital flexion contracture in a child. There are many causes of flexion contracture in the paediatric hand. Common presentations include a post-traumatic flexion contracture and camptodactyly. Upon review of the literature, there are 21 reported cases of histologically confirmed paediatric Dupuytren’s disease in the literature (Table 1) [3-21].

**Table 1:** Demographics of histologically confirmed cases of paediatric Dupuytren’s disease

Pt	Author	Age	Gender	Ethnicity	Duration	Family History	Treatment
1	Goetzee 1955 [3]	14	M	U	3 years	N	Fasciectomy
2	Hueston 1963 [4]	12	M	U	U	U	Fasciectomy
3	Rosenfeld 1983 [5]	13	F	African	3 years	U	Fasciectomy
4	Berger 1985 [6]	2	M	U	13 months	U	Segmental fasciectomy
5	Urban 1996 [7]	9	M	U	6 months	Y	Fasciectomy
6	Urban 1996 [7]	10	M	U	U	N	Fasciectomy
7	Foucher 2001 [8]	10 mo	M	U	Congenital	N	Fasciectomy
8	Rhomberg 2002 [9]	2 ½	F	U	6 months	U	Fasciectomy
9	Rhomberg 2002 [9]	10	M	U	Congenital	U	Fasciectomy
10	Mandalia 2003 [10]	10	M	U	1 year	N	Fasciectomy
11	Bebbington 2005 [11]	6 mo	M	U	U	N	Fasciectomy
12	Fernandez-Garcia 2007 [12]	12	F	U	U	U	Fasciectomy
13	Marsh 2008 [13]	8	M	U	1 year	U	Fasciectomy
14	Tiong 2009 [14]	12	M	U	18 months	Y	Fasciectomy
15	Usmar 2010 [15]	8	M	U	6 months	U	Fasciectomy
16	Korambayil 2011 [16]	4 mo	M	U	U	N	Fasciectomy
17	Kraus 2012 [17]	7	F	U	1 year	U	Fasciectomy
18	Gary 2013 [18]	6	M	Nordic	3 months	Y	Fasciectomy
19	Zheng 2013 [19]	2 ½	M	U	Congenital	N	Fasciectomy
20	Spyropoulou 2016 [20]	10	M	Greek	4 months	N	Dermofasciectomy
21	Garcia-Mata 2019 [21]	13	F	U	2 year	N	Dermofasciectomy

Dupuytren’s disease is a fibro-proliferative disease that affects the palmar fascia of the hands. It has an autosomal dominant with variable penetrance inheritance pattern. It is more common in men and those of Celtic ancestry. Not only was this case in a child, but the child was of Indian heritage and to the authors' knowledge this is the first report on a child of Indian ethnicity. Korambayil et al. have a report of paediatric Dupuytren's disease in a child of possible Indian ethnicity; however, the ethnicity is not described in their report [16]. It is classically considered a disease of adulthood and generally presents in older patients, however, can present in younger patients, particularly in those with Dupuytren’s diathesis and strong family history. It can present with a nodule in the hand and then progress to a cord-like structure with resultant flexion contracture of the digit. Skin involvement can manifest with adherence to the cord and overlying pits.

On review of the literature, there was a male preponderance (75%). Table 1 documents the demographics of the patients in all reported cases to date. In three cases, a flexion contracture was present since birth [8,9,19]. All patients presented with either a nodule or a flexion contracture. The majority of cases were treated with fasciectomy (85%). Two patients developed recurrence after simple fasciectomy and proceeded to dermofasciectomy. Urban et al. advocate dermofasciectomy as the disease can behave aggressively and recurrence can be seen early after simple fasciectomy [7]. However, recurrence was only seen after two cases in total in the literature after fasciectomy. We recommend simple fasciectomy in cases where there is no skin involvement, with dermofasciectomy reserved for recurrent cases or where the skin is also diseased, as was the case with our patient. The age of the child should be considered. If future growth spurts are anticipated, then dermofasciectomy, with the addition of skin to the digit, might reduce the risk of future scar contracture. 

## Conclusions

To conclude, paediatric Dupuytren’s disease is a rare clinical entity, particularly in a child of Indian ethnicity. Although rare, it should be included in the differential diagnosis in children presenting with flexion contractures and not just in adults. Management is similar to that of adults; however, thought should be given to the age of the child and anticipation of future growth spurts.
